The article "Functional Localizers for Motor Areas of the Brain Using fMRI" was retracted in 2023. Reasons: signs of a paper mill; compromised peer review; unreliable results or conclusions.

# Functional Localizers for Motor Areas of the Brain Using fMRI

**DOI:** 10.1155/2022/7589493

**Published:** 2022-05-28

**Authors:** Yahia Madkhali, Norah Aldehmi, Frank Pollick

**Affiliations:** ^1^Faculty of Applied Medical Sciences, Jazan University, Jizan, Saudi Arabia; ^2^College of Medical, Veterinary and Life Sciences (MVLS), University of Glasgow, Glasgow, UK; ^3^School of Psychology, University of Glasgow, Glasgow, UK

## Abstract

Neuroimaging researchers increasingly take advantage of the known functional properties of brain regions to localize motor regions in the brain and investigate changes in their activity under various conditions. Using this noninvasive functional MRI (fMRI) method makes it possible to identify and localize brain activation. There are many localizers that can be used to identify brain areas, namely, motor areas such as functional localizer, anatomical localizer, or Atlas mask. Eighteen right-handed participants were recruited for this research to test the reliability of five localizers for primary motor cortex (M1), supplementary motor area (SMA), premotor cortex (PMC), motor cerebellum, and motor thalamus. Motor execution task, namely, hand clenching was used to activate M1, SMA, and motor cerebellum. A combined action observation and motor imagery (AOMI) task was used to functionally activate PMC. Finally, a mask based on Talairach coordinates Atlas was created and used to identify the motor thalamus. Our results show that all localizers were successfully activated in the desired regions of interest. Motor execution successfully activated M1, SMA, and motor cerebellum. A novel localizer based on AOMI was successfully activated in PMC, and the motor thalamus mask obtained from the thalamus mask was successfully implemented on each participant. In conclusion, all five localizers tested in this research were reliable and can be used for rt-fMRI neurofeedback research to define the regions of interest.

## 1. Introduction

Functional magnetic resonance imaging (fMRI), a noninvasive functional imaging technique, is well known to provide high spatial resolution in imaging brain functions [1–3]. It has been widely used for functional localization and identification of brain areas in humans [4]. The use of fMRI scans to first identify brain areas of functional significance and then more closely examine the brain activity in the area is popular in neuroimaging and is known as functional localization. This approach requires conducting an independent experiment to localize the targeted region for each individual participant. Therefore, after defining the targeted region, this can then be used to analyze a task of interest in a restricted way [5, 6]. The term functional localizer refers to a functional experiment, such as fMRI, and it distinguishes this localization from anatomic information obtained from CT or structural MRI [7].

If the localizer is identified accurately, it provides a remarkable increase in sensitivity, as sensitivity decreases with a larger field of view. The anatomical constraints provided by functional localizers are used to take the form of regions of interest (ROI). These are defined operationally by reliable effects in the localizer [8].

During an experiment using a functional localizer, after ROI is determined, analysis is restricted to responses (activation) within ROI (i.e., responses averaged over voxels within ROI). As a result, there is one statistical inference; therefore, there is no need to adjust the *p* value for multiple comparisons, and responses elsewhere in the brain are ignored [9]. ROI designs, started in the late 80s in brain imaging research to define structural anatomy and receptor binding, were used, and these ROIs were used to define the characteristics of tissues of brain areas and did not identify any functional role of these areas.

These ROIs were considered useful as they showed the distribution of induced activation. However, the problem was that ROIs did not provide information about where region-specific responses are expressed [8].

Usually, functional localizer scanning is conducted separately from the main experiment. Thus, localizers introduce some inevitable confounds of both time and order. The localizer will be inappropriate if the activation pattern later changes due to time effects, for example, effects such as learning could reduce activation in some areas and increase it in other areas. The localizer scan has different aspects compared to the main experiment scan. These aspects include a number of scans, task design, and used stimuli type. This indicates that the precision with which localizing and experimental effects are estimated can be different profoundly [8, 9].

The localization of motor areas has been an objective of several research studies in the last few decades [5]. Many tools such as EEG and fMRI have been used to localize motor regions, such as M1, on the precentral gyrus. There are several fMRI-based techniques with different accuracies that have been conducted to localize motor areas in the literature, such as voluntary movement stimulation to activate regions of interest (ROI) [10, 11] and operative electrical stimulation [12, 13]. The objective of the study is to develop and test localizers for different motor areas such as M1, SMA, motor cerebellum, and motor thalamus using fMRI.

## 2. Methods

Eighteen participants were recruited for this research. They were separately recruited into three groups to test the localizer for different motor regions in the brain. All participants were right-handed, and their ages and genders are listed in Table 1.

This research has been approved by the ethics committees of the College of Science and Engineering, University of Glasgow. Each participant will provide consent for the experiment.

### 2.1. Imaging Parameters and fMRI Neurofeedback Platform

This experiment was performed in the Centre for Cognitive Neuroimaging (CCNi) at the University of Glasgow. The MRI unit is a 3T Siemens Tim Trio MRI scanner. The head coil used was a 32-channel head coil, T1-weighted image structural images were acquired using the following parameters: TR = 2000 ms; TE = 2.52 ms; 192 sagittal slices; 1 mm^3^ isotropic voxels; and image resolution, 256 × 256.

fMRI data were collected using a T2*∗*-weighted gradient echo (EPI) pulse sequence (TR = 2000 ms; TE = 30 ms; whole brain coverage with 32 axial slices; 0.3 mm gap; and 3 mm^3^ isotropic voxels).

### 2.2. First Group: Localization of Motor Regions

Twelve right-handed healthy participants were recruited to test the localizer for motor regions. This localizer aims to identify M1, SMA, and motor cerebellum. Each region was localized based on the anatomical landmark and functional localization [14]. The anatomical landmark for M1 is a sigmoidal hook or omega sign, which is a term used to denote the appearance of the hand motor area (hand knob). SMA can be defined anatomically as the area of the medial frontal cortex in the superior frontal gyrus lying dorsal to the cingulate sulcus, rostral to the primary motor cortex, and caudal to the vertical commissure anterior line [15, 15]. The cerebellum is positioned anatomically within the posterior cranial fossa of the skull, caudal to the cerebrum and tentorium cerebelli, and dorsal to the brainstem. The anterior region of cerebellum is extended interruptedly to the lateral margin of the cerebellum. The anterior region of cerebellum can be divided into the anterior lobe and the lobules simplex by the deep primary fissure [16]. Each participant underwent a high-resolution anatomical scan (T1-weighted image) and a functional localizer run.

The localizer run was composed of 7 fixation blocks (16 sec) interleaved by 6 blocks of bimanual hand clenching (30 sec).

During functional scanning of the localizer, participants were instructed either to count letters or numbers if “REST” appeared on the screen. This was carried out to control the baseline activity [17, 18]. Participants were instructed to clench their fists if “MOVE” appeared on the screen.

Functional data were preprocessed and analyzed online, with an accumulative general linear model (GLM) embedded in Turbo-BrainVoyager, and offline, using BrainVoyager. ROIs were defined in each participant in native space.

### 2.3. Second Group: Localization of the Premotor Cortex (PMC)

Three right-handed healthy participants were recruited to test the localizer for PMC.

Each participant conducted a high-resolution anatomical scan (T1-weighted image) and a functional localizer run.

The localizer scan lasts about 5 minutes, and it comprises 7 fixation blocks (16 sec each) interleaved by 6 blocks of action observation and motor imagery (AOMI) (30 sec each).

During functional scanning of the localizer, participants were instructed either to count letters or numbers if “REST” appeared on the screen and to watch videos of hand actions and imagine these actions at the same time if “Imagine” appeared on the screen. The “REST” block lasted for 16 sec, and then an “Imagine” block appeared for 30 sec. An accumulative general linear model (GLM) embedded in Turbo-BrainVoyager is used to analyze the online functional data, while BrainVoyager is used to analyze the offline functional data. ROIs were defined in each participant in native space.

### 2.4. Third Group: Localization of the Motor Thalamus

Three right-handed healthy participants were recruited in this experiment to test the localizer for the motor thalamus.

Each participant conducted a high-resolution anatomical scan (T1-weighted image) and a functional localizer run.

The thalamus was defined offline by using a thalamus mask obtained from a thalamus Atlas since we could not identify a reliable functional localizer for the motor thalamus. The thalamus mask was created offline using the Talairach Atlas [19, 20]. This mask covered motor parts of the thalamus, including ventral lateral nucleus and ventral anterior nucleus [20, 21]. This mask was used in the experimental group when the M1-thalmus connectivity was targeted. This mask was implemented individually to each participant from the anatomical scan. After implementing the mask, it was visually checked to see if it was accurately applied to localize the thalamus.

## 3. Results

### 3.1. Localization of the Primary Motor Cortex (M1)

All subjects showed activations in several areas, which are a part of the “classical” sensorimotor network, including the primary motor cortex (M1). A sigmoidal hook or omega sign, which is a term to denote the appearance of the hand motor area (hand knob), is used to identify the visual anatomy of *M*.

Figure 1 shows activation in bilateral M1 because of hand clenching. A, B, C, and D show sagittal, coronal, and transverse images of four participants.

### 3.2. Localization of the Supplementary Motor Area (SMA)

Hand clenching also introduced activations in bilateral SMA in all participants as seen in Figure 2. Panels A, B, C, and D show SMA activations in sagittal, coronal, and transverse images of four participants.

### 3.3. Localization of the Motor Cerebellum

Panels A, B, C, and D show cerebellar activation in coronal images of three participants. Red arrows indicate activation in the right anterior motor cerebellum, as seen in Figure 3. These activations include dentate nucleus, lobules IV, and lobules V.

### 3.4. Third Group: Localization of the Premotor Cortex (PMC)

All participants showed activations in the left PMC as result of AOMI. Additional activation can be seen at motor regions, such as bilateral M1. Additional activation can be seen at areas thought to be involved in motor imagery and action observation, such as SMA and visual cortex shows (Figure 4). Panels A, B, and C show sagittal, coronal, and transverse images of first, second, and third participants, respectively.

### 3.5. Third Group: Localization of the Motor Thalamus

The thalamus mask was applied on anatomical images of the participants.  Figure 5 shows the thalamus mask (red cluster) which successfully implemented on anatomical image. The anatomical image (T1 weighted image) was converted to Talairach space using BrainVoyager before implementing the thalamus mask because this mask was created based on the Talairach Atlas.

## 4. Discussion

The present study investigated aspects of localizing motor areas. First, we used motor execution of bimanual hand actions, namely, hand clenching to activate and localize M1, SMA, and cerebellum. This technique has been used widely in the field of real-time fMRI. For M1 localization, our results are in line with many rt-fMRI studies that targeted M1 for modulation using hand actions, such as hand clenching [22], fingers tapping [18, 23], and active isometric pinching [24]. These studies successfully localized M1 using localizer runs based on motor execution of actions. The precentral gyrus and the hand knob region for each participant were used to identify M1 anatomically. Functionally, M1 was localized for each participant by analyzing BOLD signals in real-time during motor execution tasks, such as hand clenching, and a square ROI was centered on the voxel with the maximal signal change during clenching relative to resting blocks. The fMRI activation signals during the hand clenching task projected into the anatomical predicted hand knob.

Then, each ROI was overlaid onto the individual's anatomical image (T1) for all participants [18].

The SMA localizer in this study successfully activated SMA because of motor execution stimuli (hand clenching). Our results are in line with [25], who used motor execution to localize SMA, and also in line with [2, 23, 26, 27], who used finger tapping as motor action to activate and localize SMA.

In addition, we used a motor execution task, namely, hand clenching, to activate the motor cerebellum. The motor cerebellum has typically been localized in previous fMRI research by implementing a cerebellum mask based on an Atlas [28]. However, previous fMRI research has also found that motor execution activates the motor cerebellum [29], especially lobules IV and V [28], and dentate nucleus [30]. Therefore, we hypothesise that a motor execution task can be used to activate the motor cerebellum to provide a functional localizer. Our results supported this hypothesis as activation was found at the cerebellum as a result of hand clenching in all participants. Therefore, this localizer is suitable for the motor cerebellum and can be used for rt-fMRI neurofeedback research targeting cerebellum modulation.

In the second group, we aimed to functionally localize PMC using a novel technique, which used action observation and motor imagery (AOMI) stimuli. According to our knowledge, this type of localizer has not been used before to localize PMC. Previous rt-fMRI research targeted PMC and used techniques to localize PMC, such as a PMC mask based on an Atlas [31, 32], motor execution [33], anatomy reference, or action observation [34]. The bilateral ventral premotor cortex and dorsal premotor cortex have all been consistently implicated in motor imagery and action observation [35]. Therefore, the idea which can be identified using AOMI stimuli [36, 37] was supported by our results. In conclusion, AOMI can be added to techniques or tasks that activate PMC, and therefore, it can be used as a localizer for fMRI studies.

In the third group, a thalamus mask was used to localize the thalamus. Since the thalamus is a deep subcortical structure, it is difficult to localize it functionally. Therefore, using a mask based on a thalamus Atlas to identify the thalamus has been used previously in fMRI studies [38, 39]. However, Liew et al. [25] used a functional localizer to identify the thalamus in their research, but they did not provide any information about the technique or task used. Here, the thalamus mask was created offline using the Talairach Atlas [19, 20]. This mask covered motor parts of thalamus including ventral lateral nucleus and ventral anterior nucleus [20]. This mask was fitted successfully individually onto each participant. Therefore, it can be used to define the motor thalamus during rt-fMRI NF research.

## 5. Conclusion

Motor execution, namely, hand clenching, can be used to functionally activate many motor areas. Our results showed that this technique successfully activated M1, SMA, and motor cerebellum functionally. Furthermore, the novel technique of an AOMI task was successfully used to functionally activate PMC. Finally, a mask of the motor thalamus was created and tested on participants, and results showed that our motor thalamus mask was accurately fitted onto each participant's anatomical image. We conclude that all localizers used in our research appeared reliable and can be used to define regions of interest for rt-fMRI research. [40].

## Figures and Tables

**Figure 1:** Sagittal, coronal, and transverse images of four participants.

**Figure 2:** SMA activations in sagittal, coronal, and transverse images of four participants.

**Figure 3:** Red arrows indicate activation in the right anterior motor cerebellum.

**Figure 4:** Sagittal, coronal, and transverse images of first, second, and third participants, respectively.

**Figure 5:** Thalamus mask (red cluster).

**Table 1:** Ages and genders of participants in each group.

	Group 1	Group 2	Group 3
Age (mean in years)	28.75	27.33	28.33
Gender	7 M, 5 F	2 M, 1 F	3 M

## Data Availability

The data used to support the findings of this study are included within the article.
